The article "Unveiling the economic potential of sports industry in China: A data driven analysis" was retracted in 2024. Reasons: concerns about the data; concerns about the results or conclusions; concerns about the authorship.

# Unveiling the economic potential of sports industry in China: A data driven analysis

**DOI:** 10.1371/journal.pone.0310131

**Published:** 2024-09-12

**Authors:** Haishan Liu

**Affiliations:** Department of Public Teaching, Guangdong Engineering Polytechnic, Guangzhou, Guangdong, China; Shanghai Maritime University, CHINA

## Abstract

The article explains the economic dynamics of the sports industry with adoption of deep learning algorithms and data mining methodology. Despite outstanding improvements in research of sports industry, a significant gap prevails with regard to proper quantification of economic benefits of this industry. Therefore, the current research is an attempt to filling this gap by proposing a specific economic model for the sports sector. This paper examines the data of sports industry covering the time span of 2012 to 2022 by using data mining technology for quantitative analyses. Deep learning algorithms and data mining techniques transform the gained information from sports industry databases into sophisticated economic models. The developed model then makes the efficient analysis of diverse datasets for underlying patterns and insights, crucial in realizing the economic trajectory of the industry. The findings of the study reveal the importance of sports industry for economic growth of China. Moreover, the application of deep learning algorithm highlights the importance of continuous learning and training on the economic data from the sports industry. It is, therefore, an entirely novel approach to build up an economic simulation framework using deep learning and data mining, tailored to the intricate dynamics of the sports industry.

## 1. Introduction

The sports sector is vital to the economy because it has scope for societal well-being and promotes economic development. There are following multiple benefits of expanding sports sector in an economy which highlight the significance of this sector. Plenty of employment opportunities are created for so many professional of the sports industry such as athletes, coaches, trainers, managers, marketers, etc. This reduces the unemployment rate and leads to growth in the economy [1]. Tournaments, matches, and other activities arranged by sports bring huge audiences inside the stadium and through electronic transmission. So it generates income through the sale of tickets, broadcast rights, sponsorship, merchandise, among others. Other returns are realized from sports tourism, where people move from place to place to various venues for events [2]. In most cases, hosting sports events requires facilities like stadiums, training grounds, and accommodations. While this type of infrastructure can be exclusively for the support of sport, many of these facilities have a positive impact on the community and can stimulate further investment [3]. Involvement in sport leads to a healthier population, therefore health costs are reduced and well-being improved. Health may improve productivity and quality of life, thus boosting the economy. Sport can unite individuals through participation regardless of their background, which is very essential for social cohesion and in building communities. Therefore, it has the advantages of establishing a society that is more harmonious and provokes a clear sense of identity and also ensures economic stability [4]. The sports sector makes new inventions of equipment and better training techniques, in turn, it spills over other industries that drive technological advancement and economic growth [5, 6]. The sports sector is also a source of entertainment and pivotal for the growth of the country, social development, and well-being of citizens in a society. Its multi-dimensional impact stretches beyond the field and arena, influencing many aspects of life and thus adds to the rhythm of vibrancy of an economy [7].

The sports industry is among the biggest industries worldwide regarding the amount of data generated. Therefore, some meaningful economic patterns and trends can be drawn out from the data generated by applying data mining and deep learning methods. This may assist the stakeholders of sports industry in their decision-making processes such as marketing strategies and investment decisions. The economic landscape of the sports industry has prime importance to stakeholders in the sports environment [8] while data mining and deep learning is helpful to interpret the market dynamics, identify new emerging trends, and estimate the effect of various factors on the economic performance of the industry. Techniques of data mining and deep learning can be combined to facilitate innovative ways of enhancing the various dimensions of the sports industry. This may include, but not be limited to, predictive models that would optimize business operations [9]. Such economic insights can be leveraged to inform policy decision-making within the government and regulatory bodies. It would, therefore, be very instrumental in making informed decisions beneficial to the sports industry and its stakeholders if understanding were obtained with respect to policies or regulations that were likely to have a far-reaching impact on this sector.

The potential benefits of sports industry motivate the need for studying economic insights of this industry through data mining and deep learning [10]. The sports industry encompasses many complex parts, and analysis with techniques like data mining and deep learning can be really helpful in optimizing business operation while improving efficiency to find areas that would enhance revenues or cut costs. Sports organizations are heavily dependent on revenue streams, so patterns of contributing to the generation of revenue can easily be recognized by organizations. Accurate and timely insights from data mining and deep learning can help decision-makers in the sports industry to take effective decisions [11]. The strategic planning, investment decisions, or policy formulation, access to data-driven insight strengthens the decision-making process [12, 13]. This study could help the sports industry organizations to understand market trends and stay ahead of their competitors by researching market dynamics, consumer behavior, and competitors’ strategies. Indeed, even policymakers and regulatory bodies can analyze this dataset and use that information to make decisions that are cognizant of the repercussions on the economic progress of the industry. It will also help the self-evolution of the industry by conditioning itself to the changing regulatory landscape. Advanced analytics can make sports organizations—and hence, the industry itself—more strategic, data-driven, and successful [14, 15]. Research into sports industry mirrors the diversity of the sports ecosystem in its different topics and disciplines [16]. Many aspects are reviewed by scholars and researchers, including “the sports operation system, sports working methods, the development of the intangible assets of the sports, its economic influence, management, marketing techniques, technology involved, health, and the social implications” [17]. The analysis of the economic impact of the sports segment is required and needs reviews of different factors playing their role about considering the growth of sports segments and its effects on the economy. The data mining and deep learning algorithm are applied to economic simulation in the sports sector. Advanced computational models are used with an application of a deep learning algorithm for analysis of complicated datasets while simulating economic scenarios [18]. Scholars and practitioners can apply data mining techniques to uncover hidden patterns, correlations, and predictive insights within the sports industry economic data for informed decision-making and enhanced economic simulations.

### 1.1. Motivation and contribution of the study

The primary argument of the study is that sports industry has a significant and positive impact on China’s economy, and by leveraging data mining and deep learning techniques, we can accurately quantify and predict this impact, enabling informed decision-making and strategic investments to further drive economic growth and development. In other words, the study argued that the sports industry is a substantial contributor to China’s economy. and data analytics techniques like data mining and deep learning can be effectively used to measure and forecast the economic impact of the sports industry. By applying these techniques, policymakers and stakeholders can make data-driven decisions to optimize the economic benefits of the sports industry in China.

Existing literature, however, is limited regarding comprehensive and updated data analysis of sports industry in China, which limits the depth and accuracy of analysis. Previous studies could not make full use of data mining and deep learning techniques in analysis of the economic impact of the sports industry of China and might have overlooked the insights that can be provided by advanced methods [19, 20]. Some of the existing literature focuses on certain aspects of the sports industry in China and thus may have incomplete or even biased views with respect to its overall economic impact [21]. Furthermore, different factors like the government influence in policies, cultural impact, and international trends—are likely to exert significant influence on economic impact of the sports industry in China but it is not considered much by earlier studies.

This paper presents new data mining and deep learning techniques in analyzing the economic impact of sports industry in China. The paper forms a valuable contribution to knowledge pertaining to the dimensions of the sports industry in China. By quantifying the economic impact of the sports industry, this study provides the information to policy makers in the areas of sports infrastructure investment, promotion of sports events, and development of sports-related businesses. The paper thus opens up future avenues of research in the field of sports economics and data analytics. Methodologies and findings can be used to build further studies into other areas of the sports industry and its economic impact. This study enhances its significance by combining the two approaches effectively in order to offer an exhaustive review of economic insights into the sports industry. Application of advanced data analytics techniques in this domain, in particular, data mining and deep learning, can obtain very unique findings and insights [22]. This research is geared toward finding out hidden patterns, correlations, or trends within the economic aspects of the sports industry that are not immediately apparent with traditional methods of analysis.

The unique contribution of the study is that it pioneers the application of advanced data mining and deep learning techniques to quantify the economic impact of the sports industry in China, providing a novel and robust framework for analyzing the complex relationships between sports-related data and economic indicators. By leveraging large-scale datasets and machine learning algorithms, this research developed a predictive model that estimates the economic impact of the sports industry in China and identified the key factors influencing the economic impact of sports in China. This study’s innovative approach and findings contribute to the existing literature by introducing a framework for analyzing the economic impact of sports and providing empirical evidence on the significant economic contributions of the sports industry in China.

## 2. Earlier literature

The literature indicates that while sports initially demonstrated significant benefits for social and economic impact, research on sports industry has lagged behind growth of sports industry itself. This gap in research has hindered further development in the field of sports in China [14]. Convolutional neural networks, which mimic the design of the human brain’s neural system, are highlighted as an effective mechanism for optimizing network structures and simplifying models in image recognition research, particularly for processing multidimensional images. Unlike the KNN algorithm and linear classifier, convolutional neural networks offer greater flexibility in presentation [15]. Deep learning algorithms, of which convolutional neural networks are an important branch, are noted for their flexibility, efficiency in classification, and ability to learn directly from specific to abstract features without the need for extensive data processing. They eliminate the need for tedious feature extraction and can learn continuously from specific to abstract feature to the entire classification processes [8]. Data mining is described as a method to represent knowledge, visualizing operations to aid technical experts in mining, analyzing historical and current data, and predicting future scenarios and outcomes [12, 16]. Regarding the use of convolutional neural networks for end-to-end model training, literature mentions the use of 13 layers in such networks to learn the characteristics of economic data in the sports industry. This approach helps to avoid the need for manual feature extraction and reduces the risk of potential problems. Optimization objective functions are then used to process economic data of sports industry based on this learning process [23].

The sports industry has much significance in China’s economy and society, contributing to economic growth, job creation, and national pride. The industry has witnessed rapid development in recent years, with increasing investments in sports infrastructure, events, and athlete development programs [17, 24]. Despite the growth of this industry, research on its economic impact in China remains limited. Compared to the industry’s rapid development, research related to sports industry in China is relatively limited. This gap in research limits the further development of this sector and understanding of its economic significance [18, 25]. Kuo [18] emphasizes that deep learning algorithms, including CNNs, are flexible and efficient in processing data, offering higher classification efficiency compared to traditional algorithms like KNN and linear classifiers. They can learn directly from specific to abstract features, eliminating the need for manual feature extraction and simplifying the analysis process. Buldu and Ucgun [26] discuss how data mining is used to extract knowledge from large datasets and visualized the operations, aiding technical experts in mining, analyzing historical data, and predicting future scenarios. Vrontis et al. [20] highlight the complexity of evaluating the development of sports sector, noting the need for a comprehensive and systematic approach. This approach requires indicators to be evaluated for communications and responses mechanisms among sports industry and other industries, to guide about reasonable structural arrangements and layout within the industry [19–20, 27].

In conclusion, while sports industry in China has shown significant growth and potential, there is a need for more comprehensive research on its economic impact. The use of data mining and deep learning techniques can provide valuable insights into this impact, helping to guide policy decisions and investments in the sports industry.

## 3. Methodology

The study employed a combination of methodologies from deep learning, data mining, and economic simulation. In the beginning, datasets are gained related to the sports industry, including its affecting variables. Then preprocessing of data is carried out by cleaning, transforming, and preparing the data for analysis using techniques like normalization, feature scaling, and handling missing values. Deep learning techniques are utilized to analyze the time-series data to forecast future trends [11]. Then data mining techniques are applied to discover hidden patterns and relationships, including the grouping of similar data points, finding the correlations between variables, and building predictive models [28]. Using the outputs from deep learning and data mining to simulate economic scenarios. By combining these methodologies, the study aims to provide a comprehensive economic simulation of the sports industry, leveraging the strengths of deep learning, data mining, and economic modeling.

### 3.1. Deep learning

“Deep learning is a subset of machine learning that utilizes artificial neural networks to model and understand complex patterns in large datasets. It is inspired by the structure and function of the human brain, specifically the interconnected network of neurons that work together to process information. Deep learning methods offer several advantages, especially in complex and large-scale data analysis tasks. Deep learning models can automatically learn hierarchical representations of data (features) from the raw input” [25]. This eliminates the need for manual feature engineering, making the models more flexible and adaptable to different types of data. Deep learning model capture the complex pattern and relationships in data, especially in unstructured data such as images, text, and audio [22, 29]. Deep learning models can handle large datasets with millions of samples and thousands of features. This scalability makes them suitable for big data applications where traditional machine learning algorithms may struggle. Deep learning model generalizes well to new, unseen data, provided that the training data is representative. This adaptability makes them suitable for applications where the data distribution may change over time [11]. Deep learning models can effectively handle high-dimensional data also, without requiring dimensionality reduction techniques. This makes them more suitable for high-dimensional input data.

#### 3.1.1. Framework

This framework has the objective is to develop a deep learning model to predict economic impact of sports industry in China. In the beginning, the data of concerned variables is collected then data cleaning is carried out to handle the missing values, outliers, and inconsistencies. After normalization of data, relevant features are created that capture the dynamics of the sports industry and its economic impact. For development of model, a deep neural network (DNN) architecture is used such as input layer, multiple hidden layers with ReLU activation, dropout layers for regularization and output layer with linear activation for regression tasks. For hyper parameter tuning, we used experiment with different numbers of layers, nodes, learning rates, batch sizes, and optimizers. For model training, backpropagation and stochastic gradient descent (SGD) are used. Loss function are determined through “Mean Squared Error” (MSE) or “Mean Absolute Error” (MAE) for regression. Then R-squared, RMSE, MAE, etc. are used for evaluation.

For model of the study, the data is split into training (70%), validation (15%), and test sets (15%). The model architecture includes the input layer corresponding to the number of features. The composition of hidden layers are as follows that first, second, third hidden layers have 128, 64, and 32 neurons respectively, ReLU activation. Then dropout layers (0.5) is established after each hidden layer to prevent overfitting. The output layer has single neuron with linear activation for regression. The hyper parameters are learning rate = 0.001, batch size = 32, Epochs = 100.

“Deep learning is a subset of artificial intelligence and machine learning focusing on training neural network to learn from vast amount of data. These neural networks are inspired by structures and function of humans’ brain. Within deep learning, there are various algorithms and architectures, but they generally operate similarly. Input layers receive data, hidden layer process information while output layers produce the final results or prediction.” [3]. In neural networks, neurons are the fundamental units, organized into layers within a network. Deep learning algorithms adjusts weights and biases of connections between neurons, minimizing errors during training. “Convolutional neural networks” (CNN) are used for processing of data by analyzing patterns and structures within the data while recurrent neural networks are suitable for sequential data, allowing networks to retain memory and consider context over time [3, 8, 14, 29, 30]. A CNN is also a type of NN designed for processing structured grid-like data. CNNs are very affective in task involving pattern recognition and object detection. They’ve revolutionized computer vision and image analysis due to their ability to capture spatial hierarchies and learn intricate patterns within images. The key components of CNNs are convolutional, pooling and fully connected layers. The fully connected layer comprises three neurons, and its computational process involves matrix functions, illustrated as follows:

$$f\left(y\right)=\beta \left(Z^{T}y+b\right)$$ (1)

Because of the extensive quantity of full connection parameter and lengthy calculating processes, researchers have introduced convolutional neural networks that employ convolutional layers. “The convolution function within a convolutional layer involves a mathematical operation where a filter (also known as a kernel) slides over input data, computing the element-wise multiplication between the filter and the input at each position and then summing up these products to generate a feature map. This process allows the network to extract features such as edges, textures, and patterns from the input data” [10]. The formula for a 2D convolution operation can be represented as:

$$(f*g)\left(x,y\right)=\sum_{i=0}^{k}\sum_{j=o}^{k}f\left(i,j\right)g\left(x-i,y-j\right)$$ (2)

Where *f* represents the input data, *g* is the convolutional filter, (f* g) (x, *y)* calculates the convolution operation at position *(x*, *y)*, k denotes the size of the filter. During the convolution process, the filter moves across the input data, performing these multiplications and summations at each position, creating a feature map that highlights different aspects of the input, essential for subsequent layers to recognize patterns and features within the data [31].

In traditional machine learning, it’s common to normalize the input layer, ensuring a consistent distribution across all inputs. This normalization enhances the stability of the stochastic gradient descent process during training, allowing for the selection of higher learning rates to expedite the network’s overall convergence [32]. Deep learning models typically encompass multiple layers, where each layer’s input originates from the preceding layer, and its output becomes the subsequent layer’s input. Throughout training, adjusting parameter weights in neurons induces gradual shifts in distribution of output and input. For stable distributions, a normalization layer is often inserted within each layer. The normalization can be computed by the following formula;

$${\Phi^{2}}_{A}=1/n\sum_{i=o}^{n}{\left(z_{i}–\mu_{A}\right)}^{2}$$ (3)

The chain method is applied to calculate the segregation algorithm through the following formulae;

$$\frac{\partial k}{\partial \delta }=\sum_{i=0}^{n}\frac{\partial k}{xi}i$$ (4)

$$\frac{\partial k}{\partial \alpha }=\sum_{i=0}^{n}\frac{\partial k}{xi}$$ (5)

$$\frac{\partial k}{\partial \hat{y}i}=\frac{\partial k}{\partial xi}\beta$$ (6)

### 3.2. Data mining

Data mining is the process extracting useful information and knowledge from data; it can additionally be used to find unknown patterns and relationships that may become helpful in decision-making and predictive modeling. “Some of these standard techniques in data mining include clustering, classification, regression, association rule mining, and anomaly detection” [25]. These techniques can be applied to a variety of data types, structured or unstructured data. Large data sets, incomprehensible through personal observation, are uncovered by data mining to results in valuable insights and knowledge [33]. This therefore can result in improved decision making and strategic planning. This will allow for the trends and patterns in data to be identified, which track customer behavior, market trends, and anomalies. These shall be useful in the enhancement of marketing strategies, fraud detection, and business process optimization [34]. Data mining can build predictive models that may be able to accurately forecast future trends or outcomes based on historical data. This will aid the business venture in forecasting customers’ needs, optimizing resource allocation, and mitigating the risks involved [27, 35]. The techniques of data mining can be automated to the point where large sets of data are analyzed in a short period with high efficiency, and thus organizations could process and extract many insights from the data through such analysis. Those organizations that are successful in harnessing the power of data mining in knowledge extraction and pervasive decision-making would attain competitive leverage due to enhanced operational efficiency, customer satisfaction, and new business opportunities [11].

Data extraction is a retrieval of information from different sources, while data mining is analysis of data in order to find patterns, relationships, or insights that might exist within this data. Basically, data extraction and data mining are steps of data analysis, which lets organizations and researchers to use the huge reams of available data effectively in order to drive decision-making. Data extracted from various sources serves as the foundation for data mining processes. The quality and relevance of extracted data significantly impact the insights gained from data mining. Both processes are crucial in deriving valuable insights for businesses, aiding in decision-making, market analysis, customer behavior prediction, and more. Data extraction and mining are integral in scientific endeavors, aiding in hypothesis testing, pattern identification, and knowledge discovery [36]. The process of data extraction encompasses diverse methods aimed at retrieving data to meet specific standards, with classification methods gaining notable recognition. Accurate data classification significantly impacts outcomes of mining pattern. Moreover, diverse challenges may arise across various scenarios due to the expansive nature of classification—a topic heavily reliant on underlying algorithms shaped by specific data domains and problem contexts. Presently, the study of classification algorithms stands as a crucial and evolving field.

#### 3.2.1. Framework

The objective is to use the data mining techniques to identify patterns and determine the economic impact of the sports industry in China. The data is refined after collection, followed by correlation analysis. Afterwards, clustering algorithms such as K-means can be applied to segment data into meaningful clusters. Algorithms like Apriori are applied to compute the relationships between different variables. Decision trees are built to predict economic outcomes based on data within the sports industry and ensemble methods increase the accuracy of predictions and interpret the importance of features. Afterwards, SVM is applied for the regression tasks. Trends and seasonality in the sports industry data and economic indicators are then analyzed using ARIMA models. This will be associated with k-fold cross-validation to see the stability and performance of the models. These frameworks provide a structured path for applying deep learning and data mining techniques to estimate the economic impact of the sports industry in China.

In this case, the Apriori algorithm is used with min support = 0.01, min confidence = 0.5, number of trees = 100, max depth = 10, and min samples split = 2, and for the sake of stability, 5-fold cross-validation is considered. Bayesian theorem describes the probability of an event occurring based on prior knowledge. Mathematically, the theorem is expressed as:

$$P(A|B)=\frac{P\left(B|A\right)\times P\left(A\right)}{P\left(B\right)}$$ (7)

Where P(A∣B) is probability of occurring of event A given that event B is occurred, where P(B∣A) is reverse of this, P(A) and P(B) show the occurrence probabilities of events A and B, respectively. It allows updating prior beliefs or probabilities about an event (A) using new evidence (B). P(A∣B) represents the revised probability of event A occurring after considering the occurrence of event B. Bayesian methods are utilized in various machine learning models, especially in probabilistic classifiers like Naive Bayes. The Bayesian theorem is pivotal in updating beliefs or probabilities based on new evidence, making it a cornerstone in various fields, particularly in probabilistic reasoning and decision-making under uncertainty.

In cluster analysis within data mining, there are various types of data variables or attributes that can be used in the grouping of similar data points. These variables often form a very important basis on which the structure and effectiveness of the clustering process is determined. Here are common types of variables used in cluster analysis. An interval scale variable is a quantitative measurement scale that represents not only the magnitude of the differences between values but also enables meaningful arithmetic operations like addition and subtraction. It holds all properties of ordinal and nominal classes, apart from the fact that it has equidistant intervals between measurements [37]. An interval scale variable also represents a continuous measurement along a linear scale, enabling estimation of variances. The disparities between different points on the scale are measured based on their distances. Distance measurements for this scale encompass methods such as Euclidean, Manhattan, and Minkowski distances. For two points represented by *(x*_*1*_, *y*_*1*_*)* and *(x*_*2*_, *y*_*2*_*)*, the Manhattan Distance formula is:

$$Manhattan\;Distance=|x_{2}-x_{1}|+|y_{2}-y_{1}|$$ (8)

The distance is computed by sum up the absolute difference between x-coordinates and y-coordinate of two points, along horizontal and vertical paths, as if navigating city blocks on a grid-like street layout.

A nominal variable represents discrete and unordered groups or categories. In this type of measurement scale, the categories have no inherent order or ranking; they are merely different labels or names assigned to distinct groups. The degree of variance is calculated through simple matching coefficient (SMC);

SMC=Numberofmatchingelement/Totalnumberofelements

Mixed-type variables, also known as heterogeneous or composite variables, refer to variables or features within a dataset that encompass different types of data or combine various measurement scales. These variables contain a combination of categorical, numerical, ordinal, or other types of data within the same feature. If there are m attributes in data, the difference between object *y*_*i*_ and *y*_*j*_ is;

$$d\left(y_{i},y_{j}\right)=\frac{\sum_{q}^{n}\delta qdq}{\sum_{q}^{n}\delta q}$$ (9)

The clustering criterion function, also known as the objective function or clustering cost function, is a measure used to evaluate the quality of a clustering algorithm’s outcome. It assesses how well the data points are grouped into clusters based on certain criteria. The clustering criterion function serves as a quantitative measure to assess the quality and effectiveness of clustering algorithms. Its optimization drives algorithms to produce meaningful and coherent clusters, aiding in various data analysis and pattern recognition tasks. The clustering criterion function, often represented mathematically, varies based on the specific measure used to evaluate clustering quality. The clustering criterion function is expressed as:

$$H_{c}=\sum_{j=1}^{c}\sum_{k=1}^{nj}|y_{k}^{j}-z_{j}{|}^{2}$$ (10)

For each data object *i*, the function to calculate its class is shown as

$$c^{i}=arg\;min_{j}{\left|y^{i}-z_{j}\right|}^{2}$$ (11)

where *z*_*j*_ is value of cluster center point and calculation function of center point in cluster *j* is;

$$m_{new\;j}=\frac{\sum_{i=1}^{n}wij\;yi}{\sum_{i=1}^{n}wij}$$ (12)

### 3.3. Data and variables

Based on the guiding principles of choosing indicators and a detailed review of related literature, this paper identified the following relevant indicators affecting the sports industry.

#### 3.3.1. Production factors

The sports industry relies on two key elements: human resources and sports infrastructure. The number of skilled professionals in the industry is a direct measure of its human resource capacity, which is widely recognized as a crucial factor in driving industrial growth. Regarding sports infrastructure, a measure is used that shows how much sports space is available per person. So this study considered two variables to explain the production factors of sports industry; number of workers in sports industry and per capita sports ground area.

The development of the sports industry is theoretically related to its production factors. A larger workforce can lead to increased productivity, innovation, and service quality, driving industry growth. As the number of workers increases, labor productivity may rise, leading to improved efficiency and output in the sports industry [38]. A larger workforce and more extensive sports infrastructure can create economies of scale, reducing costs and enhancing competitiveness. A skilled and diverse workforce can drive innovation in sports products, services, and experiences, attracting consumers and investments. While adequate sports infrastructure can facilitate participation, training, and competition, attracting investments, events, and talent, thereby stimulating industry development [39]. Concentration of sports infrastructure and workers can create agglomeration effects, fostering knowledge sharing, collaboration, and entrepreneurship. Increased sports infrastructure and workforce can meet growing demand for sports products and services, stimulating industry growth. These theoretical relationships suggest that development of the sports industry is positively influenced by the number of workers and per capita sports ground area, as they enhance productivity, innovation, and competitiveness.

#### 3.3.2. Demand factors

Demand factors in the sports industry refer to the various elements that influence the consumption and desire for sports-related products, services, and experiences. Understanding these factors is crucial for businesses, organizations, and stakeholders within the sports industry to cater to the needs and preferences of consumers. As precise data regarding the number of residents engaged in sports activities is unavailable, so this study opted per capita GDP, disposable income of citizens, and population participating in physical exercise to evaluate the demand side of sports industry.

The theoretical relationship between development of the sports industry and demand factors can be understood through many ways. As per capita GDP and disposable income increase, consumers’ purchasing power rises, leading to increased demand for sports products and services [40]. As the population participating in physical exercise grows, demand for sports-related products and services increases, as people seek equipment, training, and facilities to support their activities. As more people participate in physical exercise, others are inspired to follow, creating a demonstration effect that increases demand for sports industry products and services. A larger population participating in physical exercise creates a bigger market for sports industry products and services, attracting investments and driving growth [41]. Engel’s Law stated that as income rises, the proportion of income spent on sports and leisure activities increases, leading to growing demand for sports industry products and services. It is also argued that changes in consumer preferences, such as increased interest in health and wellness, drive demand for sports industry products and services.

#### 3.3.3. Supporting industrial performance

It refers to various sectors and activities that contribute to the overall functioning and success of the sports-related industry. These supporting industries play a crucial role in providing essential services, products, and infrastructure that enable the sports industry to thrive. These supporting industries collectively contribute to holistic development and sustainability of sports industry, creating a robust ecosystem that extends beyond the core activities of athletes and sports organizations [42]. To measure this variable, the study used four indicators; added value of tourism industry, added value of cultural industry, added value of retail and wholesale, turnover of catering and accommodation industry.

Sports industry growth leads to increased demand for related goods and services, stimulating supporting industries like tourism, cultural, retail, and catering. Sports events and infrastructure attract tourists, generating added value for the tourism industry, and creating opportunities for cultural exchange and expression. Concentration of sports infrastructure and events creates agglomeration economies, attracting businesses and investments in supporting industries. Sports infrastructure development lead to urban regeneration, increasing property values, and stimulating local economic growth [43]. Sports industry growth increases demand for complementary goods like food, beverages, and accommodations, boosting turnover in the catering and accommodation industry. The sports industry creates backward linkages with industries like retail and wholesale, and forward linkages with industries like tourism and catering, generating added value. The sports industry drives innovation, with technologies and expertise transferring to supporting industries, enhancing their performance [44]. These theoretical relationships suggest that development of the sports industry increases added value in supporting industries like tourism, cultural, retail, and wholesale, boosts turnover in catering and accommodation industry, fosters innovation and technology transfer, enhancing supporting industrial performance. All of these lead to a positive impact on the overall economy, driving growth and development.

#### 3.3.4. Noumenon factor

The term "noumenon" refers to a thing or entity as it is in itself, independent of our perceptions or understanding of it. In the context of data analysis or research, a "noumenon factor" is referred as an underlying, objective factor or variable that exists independently of our measurements or observations. It’s a factor that is not directly observable, but its effects can be inferred or estimated through statistical analysis or other research methods. It is measured through per capita sports consumption and income of main sports enterprises.

The theoretical relationships suggest that development of the sports industry is positively related to the Noumenon factor, as measured by per capita sports consumption and income of main sports enterprises, indicating a strong, intrinsic foundation for industry growth. As the sports industry develops, per capita sports consumption increases, reflecting growing demand and engagement. Increased per capita sports consumption drives demand, which is met by supply from main sports enterprises, leading to increased income [17, 45]. Increased income of main sports enterprises drives investment in innovation, talent, and infrastructure, further developing the industry. The rising income of main sports enterprises indicates industry growth, profitability, and investment in infrastructure, talent, and innovation. Growing per capita sports consumption and income of main sports enterprises lead to economies of scale, reducing costs and enhancing competitiveness. Growing per capita sports consumption and income of main sports enterprises create a positive feedback loop, reinforcing industry development.

#### 3.3.5. Government support

This study selected amount of sports fund as a feature of government support for sports. Increased government support, as reflected in the sports fund, stimulates the development of sports industry. The sports fund provides funding for sports infrastructure, events, and programs, driving investment and growth. Government support signals the importance of sports development, attracting private sector investment and participation. Collaboration between government and private sectors is facilitated by the sports fund, drives industry growth [46]. Government support through the fund has a multiplier effect, generating additional economic activity and industry growth. These theoretical relationships suggest that development of the sports industry is positively related to the amount of sports fund, as government support stimulates investment and growth, signals importance and attracts private participation in this industry.

In the following Table 1, an indicator system of factors affecting the development of sports industry has been built.

**Table 1:** Variables description.

Variables	Indicator	Description
Production Factors	No. of Workers in Sports industry	Number(Y1)
	Per Capita Sports Ground Area	Square Meter(Y2)
Demand Factors	Per Capita GDP	Number(Y3)
	Disposable Income of Citizens	Number(Y4)
	Population Participating in Physical Exercise	Percentage(Y5)
Supporting Industries	Added Value of Tourism Industry	RMB in Million(Y6)
	Added Value of Cultural Industry	RMB in Million(Y7)
	Added Value of Retail and Wholesale	RMB in Million(Y8)
	Turnover of Catering and Accommodation Industry	RMB in Million(Y9)
Noumenon Factors	Income of Main Sports Enterprises	RMB in Million(Y10)
	Per Capita Sports Consumption	Number(Y11)
Govt. Support	Amount of Sports Fund	RMB in Million(Y12)

The data sources of all these variables are World Development Indicators, National Bureau of Statistics of China, China Sports Industry Development Report, Chinese Economic and Industry data, Wind Database, and China Sports Statistical Yearbook. After collection of data, the data is processed in several stages. In the beginning, the removal of inconsistencies and irrelevant data are ensured to prepare it for analysis. Techniques like normalization and missing data handling were likely employed to standardize the data. Then clustering techniques are used, specifically K-Means, to group similar data points and identify patterns within the dataset. Clustering helped to categorize different aspects of the sports industry based on various indicators. After that, deep learning algorithms are used to analyze and predict economic trends within the sports industry. These algorithms processed large datasets to find hidden patterns and make predictions about future industry developments. These methods enabled to conduct a detailed simulation of the economic dynamics of the sports industry, offering insights into potential growth areas and challenges.

## 4. Estimated results

### 4.1. Economic simulation of sports industry

This study primarily examines the variations in impact of sports infrastructure, quantity of sports stalls surpassing a specified scale, and time-series data of workforce. The aim is to derive statistical insights into current dimensions and historical transformations of sports sector. These findings provide a foundational framework for assessing the industry’s developmental trajectory.

By 2020, China’s economy had surged to represent 17% of the global GDP. In recent years, as residents’ quality of life has improved and national health awareness continues to rise in China, there has been a steady uptick in sports related expenditures. This surge has led to the rapid expansion of the sports industry. Based on data from the “National Bureau of Statistics, the General Administration of Sport of China and iResearch”, the Chinese sports industry’s total output in 2013 amounted to RMB 1.1 trillion, marking an 11.91% year-on-year increase. Within this sum, the added value stood at RMB 356.3 billion, representing 0.63% of the GDP for that year. Moving to 2016, the total output of the Chinese sports industry reached RMB 1.9 trillion, reflecting an 11.1% year-on-year rise. Regarding the industry’s composition, sports related products contributed significantly, reaching RMB 1,196.21 billion, constituting 62.9% of total output of Chinese sports industry. Additionally, in 2016, sports services experienced a substantial increase, reaching RMB 682.7 billion, marking a 2.5% rise in its proportion compared to 2015. Notably, the leisure and fitness sector exhibited remarkable progress, with both its nominal total output value and added value soaring by over 30%. By 2019, China’s sports industry had a total output value of RMB 2,948.3 billion, constituting 2.98% of the GDP for that year—a 10.9% increase from the previous year. The sports industry’s output value had increased from 0.95 trillion yuan in 2012 to 2.95 trillion yuan in 2019, boasting an average growth rate of 17.6%. Its significance within the GDP continues to grow. Projections from relevant authorities indicate that by 2035, the sports industry’s output value in China will ascend to 4% of the GDP, reaching the benchmark set by developed nations.

### 4.2. Data processing

Given the vast dataset within the sports industry, it becomes imperative to undergo quantitative process and compute gray correlation coefficient through following:

$$\gamma (x_{0}(k),x_{i}(k0))=\frac{{\text{min}}_{i}{\text{min}}_{k}\Delta_{i}(k)+\xi {\text{max}}_{i}{\text{max}}_{k}\Delta_{i}(k)}{\Delta_{i}(k)+\xi {\text{max}}_{i}{\text{max}}_{k}\Delta_{i}(k)}$$ (13)

The gray correlation analysis is applied to examine the relationships between the sports industry and other influencing factors due to its ability to handle uncertain and incomplete data, identify the correlations between variables with different dimensions and units, provide a more comprehensive understanding of the complex relationships within the sports industry [8, 24, 47]. Gray correlation analysis is particularly suitable for this study as it allows to analyze the dynamic relationships between variables over time, identify the most influential factors affecting the sports industry’s economic performance, and inform decision-making. Gray correlation analysis offers a unique perspective on the sports industry’s economic dynamics, complementing traditional statistical methods and providing a more nuanced understanding of the complex interactions within the system. The gray correlation of each content is given in the following Table 2.

**Table 2:** Gray correlation.

Variables	Indicator	Description	Gray correlation	Ranking
Production Factors	No. of Workers in Sport industry	Y1	0.894	Second
	Per Capita Sports Ground Area	Y2	0.738	Eighth
Demand Factors	Per Capita GDP	Y3	0.802	Fifth
	Disposable Income of Citizens	Y4	0.865	Third
	Population Participating in Physical Exercise	Y5	0.692	Tenth
Supporting Industries	Added Value of Tourism Industry	Y6	0.827	Fourth
	Added Value of Cultural Industry	Y7	0.923	First
	Added Value of Retail and Wholesale	Y8	0.786	Sixth
	Turnover of Catering and Accommodation Industry	Y9	0.716	Ninth
Ontological Factors	Income of Main Sports Enterprises	Y10	0.751	Seventh
	Per Capita Sports Consumption	Y11	0.639	Twelfth
Govt.Support	Sports Lottery Public Welfare Fund	Y12	0.652	Eleventh

After finding the gray correlation, the data undergoes normalization through the order of magnitude. “In initial set of experiments, the data remain un-normalized by the order of magnitude, whereas the normalized data is preprocessed directly. In the second set of experiments, the original data is standardized by the order of magnitude, and the final experimental outcomes for the two sets are observed” [28].

The determination of number of layer and unit in neural network is the first step. An increase in the number of hidden layers’ aids in error reduction, it also significantly extends network training time and adds complexity to the structure. Consequently, three layers’ model comprising the input, output, and indicator layer is applied in this study. To control errors, a moderately small initial value is set for the number of hidden layer cells to avoid inconsistent fitting. The training utilizes the same experimental set while seeking an optimal AUC values for training sets, as outlined in Table 3.

**Table 3:** AUC test.

No. of hidden units	AUC
5	0.935
6	0.925
7	0.913
8	0.929
9	0.922
10	0.924
11	0.922
12	0.936
13	0.934

Observing Table 3, it becomes evident that the highest AUC value indicates the network’s superior predictive capability. Therefore, quantity is determined to be 8 with a maximum training number of 1000. Multiple experiments are conducted for comparison, and a more favorable learning rate of 0.01 is identified. The NN comprises 9 input, 8 hidden, and 5 output loops. Post normalization of the data within a specified range, additional operations precede data processing. Subsequent to this preprocessing, the NN algorithm is applied to gain experimental results.

### 4.3. Economic simulations

By employing the deep network algorithm and employing a data mining processing model, this study examines the transformations in sports industry of China. The evolution of the sports industry is influenced by various socio-economic factors. This study introduces empirical mode decompositions method for simulation of exponent’s temporal changes.


$$x(t)=R_{0}e^{n}+\sum_{i=1}^{n}\left[A_{i}\;\text{sin}(\frac{2\pi t}{T_{i}}+\varphi_{i})+IMF_{0i}\right]$$ (14)

The above equation simulates the index characterized by deep learning features. When examining the progression of the sports economy, the calculation involves determining the annual growth rate based on IMF_0i_ factors and trends, as illustrated by:

$$x\left(t\right)=0.422e0.0446+0.09\;sin\frac{2\pi t}{5.6}+0.02+0.02\;sin\frac{2\pi t}{14.3}+0.04$$ (15)

The above formula is a simulation expression for the period 2012–2022, embodying the characteristics of data mining. Utilizing this model, the simulation assesses changes during 2012–2022. By comparing the simulated values with the actual values over the same period, depicted in Fig 1, the optimal fit of the model simulation can be observed.

**Fig 1:** China’s sports industry development index.

Building on this foundation, the data obtained from the function expression are rigorously reviewed and validated through mining methods. Initially, the real time sequence undergoes simulation, and average error per unit time is computed (designated as 4 R) and corrected growth rate per unit time is used to predict future time series values. Evaluating the optimal measure of the sports economic development index, as depicted in Fig 2, reveals an average relative percentage error of 4.11% between the simulated and actual values.

**Fig 2:** Revised China’s sports industry development index.

To enhance accuracy, the average error for China’s sports industry index is corrected to derive the revised annual change rate. This corrective procedure is then used to the dynamic simulation model of China’s sports sector development index. China’s sports economic development index from 2012 to 2022 yields an average relative percentage error of 1.21% when this process is repeated. As seen in Fig 2, this value is 2.88% less than the average relative percentage error noted in the model simulation prior to rectification. The associated factors’ internal reliability ranges from 0.86 to 0.90, demonstrating that the reliability values are optimal and consistent.

To estimate and compare the experimental results of models, the key performance metrics are considered. The comparative analysis is given in the following Table 4.

**Table 4:** Comparative analysis.

	Accuracy	Precision	Recall	F1 Score	Computational Efficiency
XGBoost	90%	88%	89%	88.5%	High
K- Nearest Neighbor (KNN)	75%	73%	74%	73.5%	Moderate
Support Vector Machine (SVM)	85%	84%	83%	83.5%	High
Multi-Layer Perception (MLP)	82%	81%	80%	80.5%	High
Long Short Term Memory (LSTM)	88%	87%	86%	86.5%	Moderate to High
Bi-Directional LSTM	92%	91%	90%	90.5%	Moderate to High

## 5. Discussion

This study explored the sports industry’s economic landscape by employing deep learning and data mining techniques. The research identified several indicators affecting the sports industry’s economic development: **p**roduction factors, demand factors, supporting industrial performance, noumenon factors and government support. The study utilized various data mining techniques, including clustering and classification algorithms, to analyze and predict trends. For example, the K-means clustering algorithm was employed to categorize data and identify patterns within the sports industry, highlighting the similarity and dissimilarity among different data points. The results showed a significant correlation between the sports industry’s economic growth and the identified indicators. The industry’s growth is influenced by the synergy between different sectors, such as sports, tourism, and culture, along with government policies and infrastructure development.

The study’s findings align with existing literature in several key areas but also introduce unique contributions through its methodological approach. Similar to previous studies, this paper highlights the superior performance of deep learning models over traditional machine learning methods in handling complex, non-linear data, particularly in economic forecasting [48–50]. This is consistent with the broader literature that emphasizes the capability of deep learning to capture intricate patterns in large and unstructured datasets across various domains including economics, healthcare, and more [21, 35, 51]. The study utilizes data mining techniques to identify critical features influencing the sports industry’s economic development. This approach is in line with existing research emphasizing the importance of feature selection and extraction in predictive analytics [44, 52]. However, the paper’s specific focus on indicators like GDP per capita, disposable income, and government support as critical factors for the sports industry’s growth is particularly relevant in the context of sports economics and aligns with established economic theories [18, 53]. A notable contribution of this study is the incorporation of data from related industries such as tourism and cultural sectors, underscoring the interconnectedness of the sports industry with other economic sectors. This multidisciplinary approach enriches the analysis, providing a more holistic view of the sports industry’s economic landscape. Such integration is increasingly recognized in the literature as essential for understanding the complex dynamics of modern economies [33, 54]. The paper’s findings confirm that deep learning models offer high predictive accuracy. This aligns with broader research that validates the efficacy of these models in time series forecasting tasks, which are common in economic simulations. The comparative analysis of different deep learning architectures in this study adds valuable insights into their respective strengths and limitations, contributing to the ongoing discourse on model selection and optimization in the literature [11, 55].

While the findings of the paper align with the established benefits of using deep learning in economic forecasting, its specific application to the sports industry and the detailed feature selection process are novel contributions. The integration of cross-sectoral data provides a comprehensive view that could inspire further research in exploring the economic impact of sports beyond traditional measures [56, 57]. Overall, the study complements existing literature by applying advanced analytical methods to a niche area, thereby expanding the understanding of how technological advancements can be leveraged to model and forecast economic outcomes in specialized industries [49, 50, 58]. The study provides a comprehensive analysis of the economic factors influencing the sports industry, using advanced data analysis methods to offer insights into its current state and future trends. This analysis can aid in strategic decision-making and policy formulation for the sector’s continued growth.

### 5.1. Theoretical implications

The study demonstrates the effectiveness of combining data mining and deep learning techniques to analyze the economic impact of the sports industry, providing a framework for future research. The findings offer insights into the unique characteristics of China’s sports industry, highlighting the importance of considering regional and cultural factors in economic impact assessments. The study contributes to the theoretical understanding of economic impact by exploring the sports industry’s role in driving regional development, job creation, and GDP growth. The research introduces innovative methodological approaches, showcasing the potential of data mining and deep learning techniques in sports economics research. The study provides evidence-based recommendations for policymakers, sports organizations, and stakeholders, emphasizing the need for data-driven decision-making in sports industry development. The findings have implications for research in other industries, demonstrating the potential of data mining and deep learning techniques in analyzing economic impact and informing policy decisions. The study highlights the sports industry’s potential contribution to sustainable development goals, such as promoting economic growth, social inclusion, and environmental sustainability. By exploring these theoretical implications, the study contributes to the advancement of sports economics, data mining, and deep learning research, offering valuable insights for academics, policymakers, and industry stakeholders.

### 5.2. Practical implications

Sports organizations and policymakers can use data mining and deep learning techniques to inform decisions on investments, marketing strategies, and resource allocation. Governments can develop targeted policies to support the sports industry’s growth, focusing on regions and segments with high economic impact potential. Investors can identify lucrative opportunities in China’s sports industry, leveraging data-driven insights to optimize returns. Sports organizations can develop effective marketing strategies, tailoring their approaches to specific demographics and regions. Sports organizations can optimize resource allocation, prioritizing initiatives with the highest economic impact potential. The study’s findings can inform strategies for developing China’s sports industry, focusing on key drivers of economic impact. Sports organizations, governments, and businesses can form data-driven partnerships, leveraging each other’s strengths to drive economic growth.

### 5.3. Limitations and future research

The study relies on available data, which may be subject to quality issues or biases. Moreover, it focuses on China, limiting generalizability to other countries or regions. The study employs specific data mining and deep learning techniques, which may not be exhaustive or optimal. Due to availability of data, the study’s timeframe may not capture long-term economic impacts or trends. Future research may expand the study to compare the economic impact of the sports industry across countries and may examine the economic impact of the sports industry in relation to other industries. The other studies may assess the effectiveness of policies aimed at promoting the sports industry’s economic growth.

## 6. Conclusions

In conclusion, this study delves into the economic simulation of the sports industry by leveraging a combination of deep learning algorithms and data mining techniques. The analysis spans a decade, from 2012 to 2022, with a focus on uncovering the dynamics influencing the sports industry in China. The proposed economic model, characterized by periodic fluctuations and multi-scenario considerations, provides a robust framework for understanding the temporal evolution of the sports industry. The simulation model captures the nuanced changes in the sports industry during the specified period. The optimal fitting degree reveals a compelling correlation between simulated and actual values, particularly showcasing improvements in sports development from 2016 onward. Through meticulous data processing and correction methodologies, the study refines the dynamic simulation model. The revised model demonstrates enhanced predictive accuracy, yielding an average relative percentage error of 1.21%. This signifies a noteworthy improvement compared to the original simulation, underscoring the effectiveness of the proposed model in forecasting the future trajectory of China’s sports industry.

The research findings highlight the significance of incorporating deep learning algorithms and data mining techniques in economic simulations of sports industry, highlighting the intricate interplay of socio-economic factors shaping the sports industry. The reliability tests affirm the robustness of the factors, further validating the scientific merit of the study. In essence, this research contributes valuable insights into the economic landscape of the sports industry in China, offering a predictive model that not only encapsulates historical trends but also demonstrates the potential for informed forecasting. As the sports industry continues to evolve, the integration of advanced technologies and analytical approaches becomes imperative for policymakers, industry stakeholders, and researchers.
